# A DEA-Based Decision Support Framework for Organizations' Performance Evaluation considering TQM and Knowledge Management

**DOI:** 10.1155/2021/6654600

**Published:** 2021-04-13

**Authors:** Azin Karami, Hadi Shirouyehzad, Milad Asadpour

**Affiliations:** ^1^Department of Industrial Engineering, Najafabad Branch, Islamic Azad University, Najafabad, Iran; ^2^Department of Information Systems and Operations Management, Business School, The University of Auckland, Auckland, New Zealand; ^3^Young Researchers and Elite Club, Najafabad Branch, Islamic Azad University, Najafabad, Iran

## Abstract

Total quality management (TQM) and knowledge management (KM) play a significant role in improving the situation of the organization and creating and maintaining competitive advantage (CA). Therefore, harmonizing TQM and KM with the organizational goals and performance leads to the organization's greater capabilities. The current paper presents a decision support framework to evaluate the performance of organizations based on the success factors (SFs) of TQM and KM using the BCC model of data envelopment analysis (DEA). The SFs of KM are considered as input and the SFs of TQM are considered as output of the BCC model, and the efficiency scores of five pharmaceutical companies in Esfahan, Iran, are obtained. The results show that, among the aforementioned companies, three companies were recognized as efficient, while two of them were introduced as inefficient companies. Furthermore, in order to provide more recommendations for the managers of these companies, two area charts according to SFs of TQM and KM were drawn, and the results were analyzed and discussed.

## 1. Introduction

TQM is the art of managing an entire organization to get the best out of it. In the TQM approach, the main focus is on quality, particularly the quality of work and processes. Therefore, TQM is contrasted with result-oriented management, which only emphasizes result and more production. In general, the important principles governing TQM are the senior management's commitment, customer orientation, evaluation, and decision-making based on facts, participation and collaboration, training, and continuous improvement [1]. TQM is a smart, smooth, and continuous action that has a synergistic effect on achieving the goals of the organization and ultimately leads to customer satisfaction, increasing efficiency, and boosting the ability of competing in the market [2]. One of the main features of TQM is its ability of integrating techniques and methods which are related to management and quality issues comprehensively. Additionally, it has a close relationship with KM and performance management. Consequently, TQM's principles and attitudes underlie the gradual evolution of the learning organization, and its attitudes radically change it [3].

On the other hand, knowledge is assumed to be a strategic and intangible asset that can help organizations maintain their competitiveness in a turbulent environment [4]. KM is the success secret of organizations in the 21st century. Organizational managers can rely on superior knowledge to make more sensible decisions on important issues and improve knowledge-based performance [5]. In fact, KM is an organizational issue that seeks to control the spiritual and intangible capacities, experiences, and skills of employees. Therefore, in the increasing and accelerating enlargements era, organizations should employ novel managerial approaches to gain CA and survive in the market. However, creating new knowledge in the organization is required for most quality enhancement programs [6–10].

Companies need a TQM procedure that presents knowledge as a potential source of CA. TQM and KM play an important role in improving the situation of the organization, its long-term survival, as well as creating a CA for it. Accordingly, how to institutionalize these two important issues (TQM and KM) and harmonizing them with organizational goals and performance is important. Hence, the managers of organizations should try to create a mechanism for making a special situation for TQM and KM as fundamental rules which are accepted by employees, because successful organizations have the capacity of attracting TQM and KM as an organizational culture. Nonetheless, based on a review on previous research in the areas of TQM and KM, although the combination of DEA and TQM or DEA and KM has been used in the previous studies, any research which simultaneously investigates TQM and KM factors in performance evaluation applying a DEA approach was not observed. Also, among conducted research in pharmaceutical companies, any research which considered TQM and KM in performance evaluation concurrently was not observed. Meanwhile, since TQM and KM play an important role in providing continuous improvement and CA to all industries including pharmaceutical sector, it is vital to examine their simultaneous impact on the performance of pharmaceutical companies. Therefore, in the present study, the BCC model of DEA is applied to measure the performance of five pharmaceutical companies in Esfahan, Iran, over the period of March 2018 to September 2018, so that the SFs of KM and the SFs of TQM are considered as the inputs and outputs of the model, respectively. Besides, managerial directions based on the results of two area charts have been provided.

For this purpose, firstly, by reviewing previous research and consulting university experts, the SFs of TQM and KM were determined and, using distributed questionnaires within pharmaceutical companies in Esfahan, the importance and performance of SFs of TQM and KM were measured. The reliability and validity of the questionnaires were also investigated using Cronbach's alpha, Exploratory Factor Analysis, and Lawshe's method, respectively. Then, using data mining algorithms, the SFs of TQM and KM were clustered. Considering the clustered SFs of KM and TQM as input and output of a variable Return to Scale (RTS) model of DEA, namely, BCC model, the relative efficiency scores for aforementioned pharmaceutical companies were calculated. To sum up, the innovative contributions of this research are as follows:

- Identifying and clustering SFs of TQM in pharmaceutical companies
- Identifying and clustering SFs of KM in pharmaceutical companies
- Simultaneous usage of clustered SFs of TQM and KM for performance evaluation by deploying data envelopment analysis
- Applying the proposed approach within real pharmaceutical companies
- Providing practical suggestions and managerial insights with respect to results of implementing the proposed approach within the pharmaceutical companies

The rest of the current paper is organized as follows.

To begin, the previous related studies are reviewed, the research gap, and the research innovation is highlighted. Next, the concepts and tools are elaborated. In the methodology section, the steps of the present research are explained. After that, in the data collecting and analysis section, the collected data are prepared to enter the BCC model and performance evaluation of the pharmaceutical companies. Following this and in the managerial directions section, two area charts are presented and analyzed for the SF of TQM and KM. Finally, in the conclusion section, the most important results along with the limitations of the current paper are stated while some suggestions for future research are provided as well.

## 2. Literature Review

It seems that, among the previous studies, the most contribution is related to simultaneous consideration of TQM and KM and their relationships. Hsu and Shen [11] discussed the resemblances and differences between KM and TQM and suggested that both of them can be considered as a complement for another one. Molina et al. [12] evaluated how quality management (QM) affects knowledge transfers. The results obtained from a case study in Spain approved that different QM practices can be influenced on both internal and external knowledge transfers. Chong et al. [13] integrated TQM and KM approaches into a model to consider whether the hybrid procedure can improve the adoption of collaborative commerce or not. Daud and Yusoff [14] consider the effect of TQM criteria on KM processes in public firms. Results show that soft criteria of TQM such as human capital have more influence on KM and lead to better performance of organization. Ooi [15] investigates the connection between TQM and KM in manufacturing and nonmanufacturing companies in Malaysia from a multidimensional perspective. Findings reveal the relationship between TQM dimensions and KM dimensions. Alshatnawi and Abd Ghani [16] study the comprehension of staff within Jordan universities towards the application of TQM and KM rules. In particular, they indicate how comprehension of the connection between TQM and KM can affect performance of organization. Obeidat et al. [17] investigate the effect of KM criteria on TQM practices within Jordan banks. Results state that most KM criteria have a sharp effect on TQM practices. Alkhazali et al. [18] consider the influence of TQM, on human resource management (HRM) practices and KM strategies and their integrated impact on performance of Jordan banks simultaneously. Results show that TQM as a moderating factor along with HRM practices and KM strategies can lead to improvement of Jordan banks' performance. Abbas [19] examines the connection of KM, TQM, and corporate sustainability (CS) within manufacturing and nonmanufacturing companies in Pakistan. Results indicate that TQM affects CS dramatically while KM somehow mediates this relationship.

On the one hand, the innovation has been the subject of some hybrid research on TQM and KM. Hung et al. [20] studied the effect of organizational learning and TQM on innovative performance within a case study in Taiwan. Results show that both TQM and organizational learning affect innovative performance significantly. Honarpour et al. [21] illustrate the relation between KM and TQM and their integrated impact on innovation performing the Joint Variance Analysis method. In another study, Honarpour et al. [22] concentrate on R&D units in 190 firms of Malaysia and indicate how KM and TQM connection can affect the performance of R&D units from the innovation point of view.

On the other hand, the combination of DEA with either KM or TQM approaches has been noticed in the related literature. Kuah and Wong [23] applied a two-level DEA model for measuring the performance of Malaysian universities with regard to KM factors while Shirouyehzad et al. [24] considered the criteria of KM and safety management as inputs and customer satisfaction and accident indicators as outputs of a DEA model for performance evaluation of 12 companies in the car industry in Esfahan. In addition, Salhieh and Abu-Doleh [25] indicated the impact of TQM on banks efficiency applying a DEA-based approach. However, some research can be found which applied DEA for selecting, improving, or evaluating six sigma projects as well. For example, Hadi-Vencheh and Yousefi [26] and Wen et al. [27] applied a hybrid DEA technique to select six sigma projects whereas Azadeh et al. [28] performed a PCA-DEA approach to investigate the effect of six sigma extension on key job features in car industry.

Apart from TQM and KM, different methods and approaches have been employed by researchers for performance evaluation of the pharmaceutical companies. Kamath [29] studied the connection between intellectual capital (IC) criteria, profitability, productivity, and market valuation within pharmaceutical sector in India applying VAIC method. Also, Sharabati et al. [30] considered the connection between IC criteria and business performance using real data from Jordan pharmaceutical industry performing the structural equation modelling method. Mehralian et al. [31] studied the connection between IC indicators and profitability, productivity, and market valuation using real data from Iranian pharmaceutical industry and applying a hybrid approach including correlation, simple linear multiple regression, and ANN. Enekwe et al. [32] studied the impact of financial leverage on financial performance within Nigeria pharmaceutical industry during a determined time period. They have used descriptive statistics, Pearson's correlation, and regression for analyzing collected data.

Nevertheless, DEA technique has been used in several studies for performance evaluation of the pharmaceutical companies. Tavana et al. [33] studied public pharmaceutical firms and proposed a three-stage hybrid approach including MCDM, balanced scorecard, and two fuzzy DEA models. Fuzzy DEA models calculate the efficiency scores of the firms using operating budget, cost of goods as inputs, and market share, earnings per share, P/E ratio, sales growth, rank of liquidity, and volume of exports as outputs. Varmaghani et al. [34] used Malmquist index to examine the productivity status within Iranian pharmaceutical companies during 2000–2013. They considered total assets, capital stock as inputs, and net sales and net profit as outputs of the DEA model. Gascón et al. [35] evaluated the efficiency of 37 large pharmaceutical laboratories during 2008–2013 applying DEA approach. They considered employees, total assets, investment in R&D, and number of days discounted until December 13 as inputs and net income basic, market capitalization, net sales, and number of days discounted until December 13 as outputs. Al-Refaie et al. [36] applied DEA for performance evaluation of blistering lines. The planned production quantity in units, defect quantity in units, and idle time in units were considered as inputs while the actual produced quantity was the output of DEA model. Alam and Rastgi [37] performed DEA for performance evaluation of five pharmaceutical firms in India. Net block, cash and bank balance, share capital, reserve and surplus, secure loan, and unsecured loan were considered as input and investments, loans, and advances were outputs of the DEA model. Liu and Lyu [38] performed a dynamic network DEA model for evaluating the innovation efficiency of the pharmaceutical firms in China considering knowledge innovation and commercialization.

According to the above-mentioned studies, whilst the hybridization of DEA and TQM or DEA and KM has been used in the previous works, any research which simultaneously investigates TQM and KM factors in performance evaluation applying a DEA perspective was not observed. Also, among conducted research in the pharmaceutical companies, any research which considered TQM and KM in performance evaluation was not observed concurrently. Consequently, due to the existing research gap and the importance of this issue, in the present study, a DEA-based decision support framework has been presented to evaluate the performance of organizations based on the SF of TQM considering KM approach within pharmaceutical firms in Esfahan, Iran. The proposed decision support framework can provide invaluable suggestions to managers to improve their organizations' performance.

## 3. Concepts and Methods

In this section, the concepts and methods which have been applied in the present study are explained briefly.

### 3.1. TQM

TQM is a systematic structure that emphasizes the continuous improvement of all activities within an organization. In fact, TQM focuses on improving the quality of products and services by improving human resources, processes, and existing equipment, as well as reducing operating costs [39]. In other words, TQM emphasizes design, technology, and appropriate production processes selection, quality training, improving employees' involvement, considering customer requirements, and the necessity to measure the work. TQM is not just about the product; rather, it is a comprehensive view towards both the organization and the product and includes all the activities, processes, and details of the work [40]. There are different definitions for TQM which are partly presented in Table 1.

### 3.2. KM

KM deals with the management of individual and organizational knowledge in organizations to gain CA. Knowledge is a source of CA because it provides intangible assets which are unique and cannot be imitated [45]. Achieving this CA depends on the organization's ability of effectively using existing KM for creating new knowledge assets and acting based on them. Although KM seems to be a business approach, every organization should develop its own strategies to acquire the potential values of KM [46]. KM has been defined from different perspectives which are partly presented in Table 2.

### 3.3. DEA

DEA is a nonparametric performance evaluation method that was firstly introduced by Charnes et al. [52]. In fact, they generalized Farrell's [53] single-input single-output technical efficiency measure to the multiple-input multiple-output case to evaluate the relative efficiency of peer units with respect to multiple performance measures [54–57]. The units under evaluation in DEA are called decision-making units (DMUs) and a DMU is considered to be efficient when no other DMU can produce more outputs using an equal or lower amount of inputs [58–60]. What makes the difference in DEA models is the concept of RTS. In the case of constant RTS, the CCR model will be used. Meanwhile, in terms of variable RTS, the BCC model should be used. Since recognizing the RTS is a long-term procedure, there is a need to collect data from different periods and analyze them [61], and regarding the limitations on data collection (we only were allowed to collect data in one period) we were not able to determine the RTS. Consequently, by consulting with related experts, both university experts and specialists in pharmaceutical companies, we assumed that RTS is variable. As a result, in this research, under this assumption that the RTS is variable, a BCC model is performed. It should be noticed that, in both input-oriented and output-oriented DEA models as well as envelopment and multiplier DEA models, efficient DMUs would be the same. In other words, there is no difference in the recognized efficient DMUs in all aforementioned modes of BCC model. Thus, we have used the envelopment input-oriented BCC model in this research. The applied model is as follows [62–64]:

(1) $$\begin{array}{c} \text{Min}\theta \\ s.t\\ \overset{n}{\underset{j=1}{\sum }}\lambda_{j}x_{ij}\leq \theta x_{ip}\;i=1,2,\ldots m\\ \overset{n}{\underset{j=1}{\sum }}\lambda_{j}y_{ij}\geq y_{rp}\;i=1,2,\ldots m\\ \sum_{j=1}^{n}\lambda_{j}=1\\ \lambda_{j}\geq 0\;j=1,2,\ldots ,n\\ \theta \text{Free}. \end{array}$$

## 4. Methodology

First of all, the SFs of TQM and KM are extracted from reputable scientific references and library studies and will be selected according to the opinions of university experts who are faculty members. Accordingly, academic experts selected the 14 factors identified by Talib et al. [65] as SFs of TQM and the 12 factors recognized by Valmohammadi and Ahmadi [66] as SFs of KM. In the next step, based on identified indicators in the previous step, questionnaires are distributed among experts of pharmaceutical companies to collect required data. In the DEA, if the number of DMUs is considerably less than the number of inputs and outputs, then the number of efficient units will increase and consequently the obtained efficiency scores will not be valid. Since, in this study, there are five DMUs (pharmaceutical companies) which are lower than the total number of inputs and outputs (12 factors for KM and 14 factors for TQM), therefore, an appropriate data mining method is employed to reduce the number of inputs and output criteria. Next, to calculate the efficiency scores for pharmaceutical companies, an appropriate DEA model (with respect to variable RTS) is applied and companies are categorized as efficient and inefficient companies. Also, complementary explanation and analysis are provided through two area charts. It should be mentioned that, among six pharmaceutical companies in Esfahan, Reyhaneh Pharmacy did not agree to share its data in this study. Therefore, this study was conducted using collected data from five other pharmaceutical companies in Esfahan.

The steps of this research are summarized as follows:

1. Identifying the SFs of TQM and KM
2. The SFs of TQM and KM are identified according to a comprehensive review on related previous works and consultation with university experts.
3. Measuring the importance of SFs of TQM and KM
4. The importance of the mentioned factors is measured using the relevant questions in the researcher-made questionnaire of TQM and the researcher-made questionnaire of KM which are filled by experts of pharmaceutical companies.
5. Measuring the performance of SFs of TQM and KM
6. The performance of the mentioned factors is measured using the relevant questions in the researcher-made questionnaire of TQM and the researcher-made questionnaire of KM which are filled by experts of pharmaceutical companies.
7. Clustering the key SFs of TQM and KM
8. For this purpose, the K-means algorithm and the SPSS software are applied.
9. Calculating the relative efficiency of pharmaceutical companies
10. Clustered SFs of KM and TQM are considered as inputs and outputs of the BCC model and the relative efficiency is calculated for pharmaceutical companies.
11. Providing managerial directions
12. This step is done by drawing two area charts for SFs of TQM and KM.

Figure 1 depicts the steps of the present study.

## 5. Data Collection and Analysis

In this section, the procedure of data collection, the selection of SFs of TQM and KM, the method of clustering SFs of TQM and KM, and ultimately the efficiency calculation of all pharmaceutical companies are elaborated in detail.

### 5.1. Identifying the SFs of TQM and KM

After a detailed literature review and with respect to the academic experts' suggestions, 14 SFs identified by Talib et al. [65] for TQM and 12 SFs recognized by Valmohammadi and Ahmadi [66] for KM were selected.  Table 3 contains SFs of TQM identified by Talib et al. [65].

Also, Table 4 includes SFs of KM identified by Valmohammadi and Ahmadi [66].

### 5.2. Measuring the Importance of SFs of TQM and KM

Using a researcher-made questionnaire, including 71 questions related to the SFs of TQM, the importance of 14 identified SFs of TQM is measured by experts of pharmaceutical companies in Esfahan, including managers, supervisors, and specialists based on the five-point Likert scale. Finally, according to 14 questions related to the importance coefficient of these factors in organizations and using averaging, the importance of each of the SFs of TQM is determined for each firm.  Table 5 contains the results of the completion of the questionnaire by 58 experts of pharmaceutical companies in Esfahan for the importance of the SFs of TQM.

Also, through performing a researcher-made questionnaire, including 69 questions related to the SFs of KM, the importance of 12 identified SFs of KM is measured by experts of pharmaceutical companies in Esfahan, including managers, supervisors, and specialists based on the five-point Likert scale. Finally, according to 12 questions related to the importance coefficient of these factors in organizations and using averaging, the importance of each of the SFs of KM is determined for each firm.  Table 6 depicts the results of the completion of the questionnaire by 58 experts of pharmaceutical companies in Esfahan for the importance of the SF of KM.

### 5.3. Measuring the Performance of SFs of TQM and KM

To measure the performance of each of the SFs of TQM, 57 remaining questions in the researcher-made questionnaire for TQM are answered by experts of pharmaceutical companies based on the five-point Likert scale. Consequently, according to these questions and using averaging, the performance of each of the SFs of TQM is determined for each firm.  Table 7 illustrates the results of the completion of the questionnaire by 58 experts of pharmaceutical companies in Esfahan for the performance of the SFs of TQM.

Furthermore, to measure the performance of each of the SFs of KM, 57 remaining questions in the researcher-made questionnaire for KM are answered by experts of pharmaceutical companies based on the five-point Likert scale. Consequently, according to these questions and using averaging, the performance of each of the SFs of KM is determined for each firm.  Table 8 reveals the results of the completion of the questionnaire by 58 experts of pharmaceutical companies in Esfahan for the performance of the SFs of KM.

### 5.4. Clustering the Key SFs of TQM and KM

In DEA models, when the number of DMUs is lower than the number of inputs and outputs noticeably, the number of efficient DMUs increases irrationally and therefore the results of the DEA model will not be reliable. In such a situation, it is necessary to somehow reduce the number of inputs and outputs. To do so, in the current study, 12 SFs of KM and 14 SFs of TQM, which are the inputs and outputs of the model, are clustered using the SPSS software and the K-means algorithm to decrease the number of inputs and outputs. During the execution of the algorithm, the factors of the same cluster will have the most similarity to each other while the factors in different clusters will not resemble.

For clustering, firstly, the number of clusters must be determined for the K-means algorithm. Hence, the SPSS software and the Hierarchical Clustering method are used. Figures 2 and 3 show the dendrogram diagram which determines the number of clusters of the SFs of TQM and KM, respectively.

In fact, after determining the number of clusters using the Hierarchical Clustering method in the SPSS software, the K-means algorithm is executed and the main SFs of TQM and the main SFs of KM are clustered into three clusters. Thus, with the implementation of this algorithm, firstly, some points are selected as the initial centralization in each dimension for TQM and KM randomly. The number of these points is selected according to the number of clusters that were determined in the previous step by the Hierarchical Clustering method, which were three clusters. Then, the closest points to each center form a cluster, and the algorithm will be repeated for other dimensions. Besides, each time the algorithm is repeated, the centrality of each cluster is iterated by averaging the factors in each cluster, and the algorithm is replicated until placing all the factors in the appropriate clusters according to their similarity. Tables 9 and 10 show the clustering results of the SFs of TQM and KM, respectively.

Ultimately, the average score of the factors related to each cluster indicates the final score of the cluster. Tables 11 and 12 show these values for SFs of TQM and SFs of KM in each organization, respectively.

### 5.5. Calculating the Relative Efficiency of Pharmaceutical Companies

To calculate the efficiency of pharmaceutical companies in Esfahan, the BCC input-oriented model is used. The clustered data of KM are considered as input of the model (three inputs) and the average of the clustered data of TQM is considered as the output of the model (one output) and the efficiency values for DMUs (pharmaceutical companies) are obtained. The inputs and outputs of the model as well as the calculated efficiency for each DMU applying the BCC model are presented in Table 13.

It should be noted that organizations with an efficiency score of 1 have the best performance and will be efficient. Accordingly, organizations are divided into two categories, namely, efficient companies and inefficient companies.

### 5.6. Managerial Directions

In this section, with the aim of explaining how the proposed decision support framework of the current paper can be helpful for managers of pharmaceutical companies, some recommendations are provided. To do so, based on measuring the value of importance and performance and the average score of SFs of TQM with KM approach, two area charts are drawn and analyzed.

In the area chart of TQM, the vertical axis is the importance average of the SFs of TQM for the five pharmaceutical companies in Esfahan (average values of each row of Table 5) and the horizontal axis is the performance average of the SFs of TQM for the aforementioned pharmaceutical companies (average values of each row in Table 7).  Table 14 contains the required data for drawing the area chart of TQM. In addition, Figure 4 presents the area chart of TQM.

In the same way, the area chart of KM is drawn for the SFs of KM. In the area chart of KM, the vertical axis is the importance average of the SFs of KM for the five pharmaceutical companies in Esfahan (average values of each row of Table 6) and the horizontal axis is the performance average of the SFs of KM for the aforementioned pharmaceutical companies (average values of each row in Table 8).  Table 15 contains the required data for drawing the area chart of KM. In addition, Figure 5 presents the area chart of KM.

As it can be seen in the area chart of TQM, SFs of TQM in the five pharmaceutical companies in Esfahan are located in the four areas of Figure 4.

  Area 1: area chart of TQM.
  Four factors including organizational culture, benchmarking, supplier relationship management, and human resource management are located in area 1. In this area, the performance values of these factors within the five pharmaceutical companies in Esfahan are lower than average whereas their importance values are greater than average. Therefore, considering the importance of TQM, five pharmaceutical companies should pay more attention to these factors. In other words, these factors have a high priority for immediate improvement.
  Area 2: area chart of TQM.
  Three factors including leadership and top-management support, organizational structure, and reward and encouragement are located in area 2. In this area, both performance values and importance values of these factors within the five pharmaceutical companies in Esfahan are higher than average. Hence, these factors are in a desirable situation in pharmaceutical companies compared to other factors. In fact, these factors provide a CA for pharmaceutical companies, and the right solution is to continue to act in the same way as before.
  Area 3: area chart of TQM.
  Three factors including TQM strategy, customer relationship management, and continuous improvement are located in area 3. In this area, both the performance values and the importance values of these factors are lower than average. Accordingly, these factors do not require any additional investment, since these factors are neither critical nor threatening for the five pharmaceutical companies.
  Area 4: area chart of TQM.
  Four factors including process management, control, and improvement, data analysis, resource innovation, and training and education are located in area 4. In this area, the performance values of the SFs of TQM within the five pharmaceutical companies in Esfahan are higher than the average while the importance values are lower than the average. Thus, pharmaceutical companies should modify the allocated resources to these factors and focus on other factors, especially those located in area 1.

Similar to the area chart of TQM, SFs of KM in the five pharmaceutical companies in Esfahan are located in the four areas of Figure 5 as well.

  Area 1: area chart of KM.
  Two factors including organizational culture and performance measurement are located in area 1. In this area, the performance values of these factors within the five pharmaceutical companies in Esfahan are lower than average whereas their importance values are greater than average. Therefore, considering the importance of KM, five pharmaceutical companies should pay more attention to these factors. In other words, these factors have a high priority for immediate improvement.
  Area 2: area chart of KM.
  Two factors including leadership and top-management support and information technology are located in area 2. In this area, both performance values and importance values of these factors within the five pharmaceutical companies in Esfahan are higher than average. Hence, these factors are in a desirable situation in pharmaceutical companies compared to other factors. In fact, these factors provide a CA for pharmaceutical companies, and the right solution is to continue to act in the same way as before.
  Area 3: area chart of KM.
  Five factors including KM strategy, reward and encouragement, training and education, human resource management, and benchmarking are located in area 3. In this area, both the performance values and the importance values of these factors are lower than average. Accordingly, these factors do not require any additional investment, since these factors are neither critical nor threatening for the five pharmaceutical companies.
  Area 4: area chart of KM.
  Three factors including organizational infrastructure management, processes and activities, and removing resource limitations are located in area 4. In this area, the performance values of the SFs of KM within the five pharmaceutical companies in Esfahan are higher than the average while the importance values are lower than the average. Thus, pharmaceutical companies should modify the allocated resources to these factors and focus on other factors, especially those located in area 1.

## 6. Concluding Remarks and Future Research

Simultaneous investigation of TQM and KM in the performance of organizations can help organizations in the continuous improvement and benefiting from the CA as much as possible, because this concurrent investigation compares organizations from TQM and KM perspectives and determines the aspects that each organization can focus on to achieve better results. Accordingly, in a long-term horizon, organizations will be able to institutionalize TQM and KM as a culture in their organization and exploit its advantages in improving the organization's performance.

In this study, we evaluated the performance of pharmaceutical companies in Esfahan considering TQM and KM using a DEA model. Initially, the SFs of TQM and KM were selected by reviewing previous studies and consulting academic experts. Then, two researcher-made questionnaires were distributed among the experts of pharmaceutical companies in Esfahan to examine the SFs of TQM and KM, respectively. Within these researcher-made questionnaires, the importance values of the SFs of TQM and KM were determined. Next, in order to evaluate the performance of organizations, the BCC model was used, so that the clustered SFs of KM and TQM were considered as inputs and outputs of the model, respectively. Among the five pharmaceutical companies in Esfahan, three companies, namely, Amin, Farabi, and Goldaru, were determined as efficient pharmaceutical companies.

In addition, in order to provide more insight towards the organization for managers, two area charts were presented for SFs of TQM and KM, respectively, and results were analyzed and discussed. Accordingly, the factors which were located in area 1 need to be improved instantly. In this group, “organizational culture,” “benchmarking,” “supplier relationship management,” and “human resource management” as the four SFs of TQM and “organizational culture” and “performance measurement” as the two SFs of KM need immediate improvement. Also, factors which were located in area 2 were in the favorable situation, and organizations need to continue applying the current procedure about these factors. In this regard, “leadership and top-management support,” “organizational structure,” and “reward and encouragement” as the three SFs of TQM and “leadership and top-management support” and “information technology” as the two SFs of KM should be retained in the current situations. Further, factors in area 3 including “TQM strategy,” “customer relationship management,” and “continuous improvement” as the three SFs for TQM and KM strategy and “reward and encouragement,” “training and education,” “human resource management,” and “benchmarking” as the five SFs of KM are factors that are not a threat to organizations and do not need to be considered. However, “process management, control, and improvement,” “data analysis,” “resource innovation,” and “training and education” as the four SFs of TQM and “organizational infrastructure management,” “processes and activities,” and “removing resource limitations” as the three SFs of KM were located in area 4. In consequence, these SFs should be reconsidered and their resources should be reassigned to the factors in area 1. Therefore, in selecting managers of different departments in organizations, it should be taken into account whether the department needs to improve or should it retain the current situation.

It is noteworthy that, among the SFs of TQM and KM in the five pharmaceutical companies in Esfahan, Jey Pharmed Spandana, and Farabi have had the highest performance in the factor of leadership and top-management support. Given that the success of any project in the organization requires the participation and support of senior managers of that organization, the style of leadership and top-management support in these two companies can be considered as a benchmark, so that if other companies implement this style within their organization, they will observe an improvement in their performance.

Apart from advantageous aspects of this research which have been highlighted within the text in detail, similar to other studies, there are limitations as well. Considering that this research has been conducted in the city of Esfahan, as one of the most developed regions of Iran, the results have been obtained according to the specific culture and social conditions of this city. However, since pharmaceutical companies are expanded across the country, caution should be exercised in generalizing the results of this research to pharmaceutical companies which are located in other cities and regions that are less developed. Also, the research findings are limited to the case study (pharmaceutical companies in Esfahan) and by changing the case, probably different results are obtained. Therefore, it is not possible to generalize the findings to other organizations. Moreover, it should be noted that, in addition to the SFs of TQM and KM which were used in this study, other factors may affect the success of TQM and KM that were not considered in this study. Another limitation of this study is that the validity of the research findings depends on the time of data collection. Therefore, if the data is collected at other intervals, it is possible that the results will change.

Because, in this study, only the questionnaire tool was used to collect data, researchers in future studies can apply different methods of interview to collect data. Performance evaluation based on the other SFs of TQM and KM can also be considered in future research. On the other hand, due to the fact that the K-means algorithm has been used in the present study, in future research, other clustering algorithms or other statistical methods can be employed to determine the relationship between variables and select input and output variables. Since the benefits of TQM and KM are not limited to the pharmaceutical companies, effects of these approaches on performance of other industries and companies could be addressed in future research. In fact, by using SFs of TQM and KM as the inputs and outputs of the DEA model, other firms and industries can enjoy our proposed framework for performance evaluation and analyze the effects of TQM and KM on their performances. Furthermore, because the data of this study were collected in a specific time period, data collection at different intervals and using other performance evaluation methods such as dynamic DEA or the Malmquist index method which consider different time intervals in data analysis could be addressed in future research.

## Figures and Tables

**Figure 1:** Research steps.

**Figure 2:** Dendrogram diagram for determining the number of clusters of TQM success factors.

**Figure 3:** Dendrogram diagram for determining the number of clusters of KM success factors.

**Figure 4:** Area chart of TQM.

**Figure 5:** Area chart of KM.

**Table 1:** Definitions of the TQM.

Author(s)	Definition
Dubey and Gunasekaran [40]	TQM is an effective cost management system for continuous efforts to improve people at all levels.
Kanji et al. [41]	It is a process that constantly satisfies the customer's needs with a reasonable cost using each person's abilities.
Harnesk and Abrahamsson [42]	TQM is a higher credit symbol.
Taddese and Osada [43]	It is a philosophy which develops the market and improves the success of the company's business.
Kristianto et al. [44]	It is a strategy to increase customer satisfaction.

**Table 2:** Definitions of the KM.

Author(s)	Definition
Davenport [47]	It is an effort to discover the hidden assets in people's minds and turn them into the organizational assets, so that this asset be accessible for all employees to exploit it.
O'Dell et al. [48]	It is a systematic procedure to finding, comprehending, and applying knowledge for value creation.
Choy and Suk [49]	It is a framework for integrating interactions at all activity levels of an organization so that the firm can use its knowledge and, if it is required, gain new knowledge for value creation for its customers and stakeholders. This managerial structure integrates individuals, processes, and technology for sustainable performance development.
Nevo and Chan [50]	It is an integrated procedure to recognize, collect, retrieve, share, and measure an organization's information capital. The information assets may include databases, documents, mechanisms, methods, or even the experiences of managers.
Karkoulian et al. [51]	It is a way for establishing an organization whose members can gain, share, and create knowledge or employ it for decision-making.

**Table 3:** SFs of TQM.

Code	Success factor
T1	Leadership and top-management support
T2	Organizational culture
T3	TQM strategy
T4	Benchmarking
T5	Organizational structure
T6	Process management, control, and improvement
T7	Data analysis
T8	Customer relationship management
T9	Supplier relationship management
T10	Reward and encouragement
T11	Resource innovation
T12	Training and education
T13	Continuous improvement
T14	Human resource management

**Table 4:** SFs of KM.

Code	Success factor
K1	Leadership and top-management support
K2	Organizational culture
K3	Information technology
K4	KM strategy
K5	Performance measurement
K6	Organizational infrastructure management
K7	Processes and activities
K8	Reward and encouragement
K9	Removing resource limitations
K10	Training and education
K11	Human resource management
K12	Benchmarking

**Table 5:** Importance values of SFs of TQM.

Code	Name of pharmaceutical company				
	Raha	Goldaru	Jey Pharmed Spandana	Amin	Farabi
T1	3.917	3.684	4.667	3.875	3.846
T2	3.667	3.921	3.417	3.938	3.846
T3	3.306	3.421	3.556	3.833	3.974
T4	3.750	3.579	4.000	3.250	4.538
T5	3.500	3.474	3.750	3.563	4.038
T6	3.467	3.263	3.567	3.450	4.200
T7	3.139	2.982	3.889	3.167	4.205
T8	3.583	3.526	3.833	3.250	3.846
T9	3.583	3.789	4.333	4.125	4.308
T10	3.467	3.589	3.833	3.525	4.376
T11	3.333	2.579	3.167	3.500	3.385
T12	3.167	3.211	3.167	3.375	3.692
T13	3.250	3.263	3.833	3.375	4.308
T14	3.750	3.579	4.000	3.250	4.538

**Table 6:** Importance values of SFs of KM.

Code	Name of pharmaceutical company				
	Raha	Goldaru	Jey Pharmed Spandana	Amin	Farabi
K1	3.917	3.737	4.500	3.857	3.923
K2	3.528	3.404	4.056	3.762	4.048
K3	3.500	3.526	4.333	3.429	4.143
K4	3.500	3.158	4.000	3.857	3.643
K5	3.583	3.421	3.833	3.571	4.429
K6	3.333	3.263	3.500	3.429	4.143
K7	3.125	3.421	3.500	3.500	3.964
K8	3.000	3.368	4.167	3.143	3.643
K9	3.083	3.368	3.833	3.571	4.214
K10	3.333	3.368	3.833	3.143	4.000
K11	3.125	3.316	4.000	3.500	4.143
K12	3.167	3.368	3.667	3.857	3.857

**Table 7:** Performance values of SFs of TQM.

Code	Name of pharmaceutical company				
	Raha	Goldaru	Jey Pharmed Spandana	Amin	Farabi
T1	3.194	2.934	3.722	3.762	3.964
T2	2.885	2.789	3.271	3.232	3.786
T3	3.194	2.711	3.194	3.69	4.071
T4	2.854	2.566	2.917	3.429	3.629
T5	3.467	2.979	3.667	4.086	3.839
T6	3.144	2.719	3.370	3.603	4.548
T7	3.194	3.211	3.222	3.952	4.022
T8	2.813	3.276	2.667	3.536	4.357
T9	3.028	3.316	3.056	3.714	4.238
T10	2.686	2.184	2.625	3.071	3.971
T11	3.367	3.358	3.933	3.343	3.625
T12	3.167	2.684	3.611	3.500	3.690
T13	3.000	3.105	3.000	3.571	3.723
T14	2.569	2.281	3.222	2.81	3.661

**Table 8:** Performance values of SFs of KM.

Code	Name of pharmaceutical company				
	Raha	Goldaru	Jey Pharmed Spandana	Amin	Farabi
K1	3.190	2.677	3.690	2.714	3.796
K2	2.906	2.704	3.104	2.500	3.848
K3	3.125	2.82	3.333	2.714	4.095
K4	2.917	2.693	3.167	2.629	3.762
K5	2.625	2.776	2.542	2.314	3.929
K6	2.883	2.842	3.067	2.971	3.971
K7	3.092	2.539	3.250	2.343	4.314
K8	2.467	1.947	2.200	2.542	3.686
K9	2.983	3.211	3.367	2.833	3.600
K10	2.681	2.658	3.167	2.595	3.905
K11	2.792	2.421	3.333	2.839	4.268
K12	3.111	2.544	3.000	3.000	3.833

**Table 9:** Clustering of SFs of TQM.

Code	Name of pharmaceutical company					Cluster number
	Raha	Goldaru	Jey Pharmed Spandana	Amin	Farabi	
	Performance values of success factors of TQM					
T1	3.194	2.934	3.722	3.762	3.964	3
T2	2.885	2.789	3.271	3.232	3.786	1
T3	3.194	2.711	3.194	3.69	4.071	2
T4	2.854	2.566	2.917	3.429	3.629	1
T5	3.467	2.979	3.667	4.086	3.839	3
T6	3.144	2.719	3.37	3.603	4.548	2
T7	3.194	3.211	3.222	3.952	4.022	2
T8	2.813	3.276	2.667	3.536	4.357	2
T9	3.028	3.316	3.056	3.714	4.238	2
T10	2.686	2.184	2.625	3.071	3.971	1
T11	3.367	3.358	3.933	3.343	3.625	3
T12	3.167	2.684	3.611	3.5	3.69	3
T13	3	3.105	3	3.571	3.723	2
T14	2.569	2.281	3.222	2.81	3.661	1

**Table 10:** Clustering of SFs of KM.

Code	Name of pharmaceutical company					Cluster number
	Raha	Goldaru	Jey Pharmed Spandana	Amin	Farabi	
	Performance values of success factors of KM					
K1	3.190	2.677	3.690	2.714	3.796	3
K2	2.906	2.704	3.104	2.500	3.848	2
K3	3.125	2.82	3.333	2.714	4.095	3
K4	2.917	2.693	3.167	2.629	3.762	2
K5	2.625	2.776	2.542	2.314	3.929	2
K6	2.883	2.842	3.067	2.971	3.971	3
K7	3.092	2.539	3.250	2.343	4.314	3
K8	2.467	1.947	2.200	2.542	3.686	1
K9	2.983	3.211	3.367	2.833	3.600	3
K10	2.681	2.658	3.167	2.595	3.905	2
K11	2.792	2.421	3.333	2.839	4.268	3
K12	3.111	2.544	3.000	3.000	3.833	2

**Table 11:** Average of each cluster for SFs of TQM.

Name of pharmaceutical company	Cluster 1	Cluster 2	Cluster 3
	T2, T4, T10, and T14	T3, T6, T7, T8, T9, and T13	T1, T5, T11, and T12
Raha	2.749	3.065	3.299
Goldaru	2.749	2.868	2.99
Jey Pharmed Spandana	3.336	3.014	3.598
Amin	3.203	3.571	3.82
Farabi	3.735	4.055	3.833

**Table 12:** Average of each cluster for SFs of KM.

Name of pharmaceutical company	Cluster 1	Cluster 2	Cluster 3
	K8	K2, K4, K5, K10, and K12	K1, K3, K6, K7, K9, and K11
Raha	3.011	2.848	2.467
Goldaru	2.750	2.675	1.947
Jey Pharmed Spandana	3.456	2.996	2.200
Amin	2.673	2.849	2.314
Farabi	4.007	3.855	4.296

**Table 13:** Efficiency scores of the BCC model.

Name of pharmaceutical company (DMU)	Input (KM)			Output (TQM)	Efficiency score
Raha	3.011	2.848	2.467	3.037	0.955
Goldaru	2.75	2.675	1.947	2.869	1
Jey Pharmed Spandana	3.456	2.996	2.2	3.316	0.998
Amin	2.673	2.849	2.314	3.531	1
Farabi	4.007	3.855	4.296	3.874	1

**Table 14:** Required data of area chart of TQM.

Code	Average of importance values	Average of performance values
T1	3.998	3.455
T2	3.758	3.180
T3	3.618	3.296
T4	3.823	3.078
T5	4.040	3.641
T6	3.589	3.498
T7	3.476	3.587
T8	3.608	3.263
T9	4.028	2.950
T10	3.758	3.390
T11	3.193	3.531
T12	3.322	3.406
T13	3.606	3.292
T14	3.823	2.969
Average	3.689	3.324

**Table 15:** Required data of area chart of KM.

Code	Average of importance values	Average of performance values
K1	3.987	3.271
K2	3.759	3.080
K3	3.786	3.194
K4	3.632	3.074
K5	3.768	3.003
K6	3.534	3.160
K7	3.502	3.233
K8	3.464	2.645
K9	3.614	3.158
K10	3.536	3.027
K11	3.617	3.065
K12	3.583	3.041
Average	3.648	3.079

## Data Availability

The data used to support the findings of this study are available from the corresponding author upon request.
